This article has been retracted.

# miR-181a Ameliorates the Progression of Myasthenia Gravis by Regulating TRIM9

**DOI:** 10.1155/2021/1303375

**Published:** 2021-12-09

**Authors:** Qiang Wang, Yunquan Liu, Shixiang Kuang, Ruozhao Li, Ning Weng, Zhichao Zhou

**Affiliations:** ^1^The Second Clinical Medical College of Guizhou University of Traditional Chinese Medicine, Guiyang 550002, Guizhou, China; ^2^Department of Neurology, Zhuji Affiliated Hospital of Shaoxing University, Zhuji 311800, Zhejiang, China

## Abstract

Abnormally activated CD4^+^ T cells are considered to be an important factor in the pathogenesis of myasthenia gravis (MG). In the pathogenesis of MG, the imbalance of proinflammatory cytokines and immune cells maintains the imbalance of immune response and inflammatory microenvironment. Studies have shown that miRNA is involved in the pathogenesis of MG. In our experiment, we extracted peripheral blood mononuclear cells (PBMCs) from MG patients and detected the expression of miR-181a and TRIM9 in PBMCs by qRT-PCR. In vitro experiments were conducted to explore the regulatory mechanism of miR-181a on target genes and its influence on inflammatory factors related to MG disease. Experimental autoimmune myasthenia gravis (EAMG) model mice are established, and the effects of miR-181a on EAMG symptoms and inflammatory factors are explored through in vivo experiments. According to a total of 40 EAMG mice that were successfully modeled, all EAMG mice showed symptoms of muscle weakness; their diet was reduced; their weight gain was slow; and even weight loss occurred. In MG patients and EAMG mice, the expression of miR-181a was low and TRIM9 was highly expressed. Bioinformatics website and dual-luciferase report analysis of miR-181a had a targeting relationship with TRIM9, and miR-181a could target the expression of TRIM9. After upregulating miR-181a or interfering with TRIM9, serum miR-181a in EAMG mice was significantly upregulated; TRIM9 was significantly downregulated; its clinical symptoms were reduced; and the expression of inflammatory factors was reduced. The study finally learned that miR-181a can reduce the level of MG inflammatory factors by targeting the expression of TRIM9 and has the effect of improving the symptoms of MG.

## 1. Introduction

Myasthenia gravis (MG) is an acquired autoimmune disease. The postsynaptic membrane of the neuromuscular junction (NMJ) is the site of its disease. When the acetylcholine receptor (AchR) on the postsynaptic membrane is destroyed, the number of this receptor decreases, leading to the occurrence of myasthenia gravis [1]. The body's immune system plays an important role in the pathogenesis of myasthenia gravis. Skeletal muscle is the main organ involved in myasthenia gravis, and other organs can also be affected by it. The skeletal muscles are prone to fatigue and fluctuating changes, aggravated after exercise, but the symptoms can be relieved after rest or drug treatment. Symptoms of muscle weakness are usually light in the morning and heavy in the evening. The course of the disease is chronic and protracted. Most patients have recurring attacks. The most serious consequence of the disease is muscle weakness crisis. When the respiratory muscles are affected, it can lead to respiratory failure and life-threatening [2]. It has been reported that the prevalence of MG is (77–150) per 100 thousand, and the annual incidence is (4–11) per 1 million. This disease can occur in any age group, but a large number of clinical studies have found that 20–40 years old and 40–60 years old are the two peak incidences of myasthenia gravis. MG patients between the ages 20 and 40 are more common in women, and the onset of men is between 40 and 60 years. Between the onsets, children have fewer incidences of only 10% [3, 4]. However, medical experts at home and abroad have discovered in clinical practice in recent years that the incidence of myasthenia gravis in the elderly is also gradually increasing.

The cause of the disease is still unclear. It is believed that the initial link of the disease may be environmental and genetic factors [5]. Among them, irrational use of drugs and viral infections play an important role in environmental factors; the immune genetic factors vary from person to person, mainly depending on human T cell receptors, leukocyte antigen (HLA) alleles, and so on. [6]. Its pathogenesis also needs further research and exploration by experts and scholars. With the further development of scientific research, experts and scholars at home and abroad have gradually focused on cytokines. Long-term animal experiments and clinical studies have found that factors such as interleukin-4 (IL-4), interleukin-6 (IL-6), and tumor necrosis factor-*α* (TNF-*α*) play an important role in the pathogenesis of EAMG [7, 8]. MG is generally considered to be an autoimmune disease that occurs in individuals carrying certain susceptibility genes, triggered by environmental factors. It is common for MG to coexist with other immune-mediated diseases, such as rheumatoid arthritis and thyroid disease; this also suggests that MG may be caused by the interaction between genetics and the environment. The miRNA plays a key role in the regulation of the pathogenesis of MG. miRNA is considered to be related to the immune regulation activation mechanism, especially related to the process of T cell response, inflammatory response, and the expression of inflammatory factors. The related research of MG-specific miRNA can provide value for its pathogenesis and treatment [9–11].

Studies have shown that in the pathogenesis of MG, MiR-181a can regulate the activation and differentiation of CD4^+^ T cells by targeting IL-2 [12]. TRIM9 has been thought to be related to the development of MG mice [13]. Therefore, in this study, we extracted peripheral blood mononuclear cells (PBMCs) from MG patients to detect the expression of miR-181a and TRIM9 in PBMCs. In vitro experiments were conducted to explore the regulatory mechanism of miR-181a on target genes and its influence on inflammatory factors related to MG disease. Experimental autoimmune myasthenia gravis (EAMG) model mice have been established, and the effects of miR-181a on EAMG symptoms and inflammatory factors have been explored through in vivo experiments. The specific report is as follows.

## 2. Experimental Materials and Methods

### 2.1. Clinical Samples

From June 2017 to September 2020, peripheral blood samples of 46 MG patients who met the enrollment criteria and 46 matched healthy controls were collected from this hospital. Fresh peripheral blood anti-coagulant specimens were taken and added with an equal amount of Hank's solution and mixed well. The layered solution was added to a test tube, and the amount was about 1/2 of the blood volume. Straw was used to slowly add blood to the layered liquid surface along the tube wall. It was centrifuged in a horizontal centrifuge at 1,500 r/min for 10 min. It can be seen that the vast majority of PBMCs were suspended at the interface between the plasma and stratified fluid, showing a white film shape. The cell layer at the interface was sucked with a sharp pipette and placed in another test tube, and an appropriate amount of Hank's solution was added. After mixing, the mixture was centrifuged at 1,000 r/min for 10 min, and the supernatant was discarded. Cells were resuspended in RPMI-1640 culture medium and frozen in a −90°C refrigerator for later use.

The diagnostic criteria for myasthenia gravis were a combination of the patient's clinical manifestations, electrophysiological detection of abnormal single-fiber EMG, abnormally repeated electrical nerve stimulation, and current response to treatment. Abnormal levels of anti-AChR and anti-MuSK antibodies supported the diagnosis of myasthenia gravis; however, the serum-negative antibody level did not mean that it did not meet the diagnosis of myasthenia gravis. Exclusion criteria include: suffering from cardiovascular disease and cerebrovascular disease, suffering from cognitive disease, pregnant women, other diseases that cause muscle weakness, patients with tumors other than thymoma, subjects who cannot provide informed consent, and before the study patients using immunosuppressive agents within six months.

### 2.2. Experimental Animals

There were 70 healthy and clean C57BL/6 female mice, 1 week old (8–10 weeks) and weighing about 16–20 grams (purchased from Beijing Weitong Lihua Biological Co. Ltd.). All experimental animals were fed with single-cage pellet feed in the central laboratory animal room where the hospital is located. The room temperature is maintained at 20 ± 5°C; the humidity is maintained at 40–60%; and good ventilation is maintained. Plasma water, feed, and padding needed to be replaced regularly during the breeding process. All mice were adaptively fed for one week.

### 2.3. Experimental Steps

#### 2.3.1. Grouping of Mice

Sixty mice were weighed and numbered, and the mice were divided into two groups according to the random number table method: a normal group and a model group. Eight mice in the normal group were fed normally without any manipulation; 62 mice in the model group were established for the EAMG model.

#### 2.3.2. Preparation of Immune Antigen

According to the method of Baggi et al. [14], 2.5 mg rat-derived peptide (Shanghai Gill Biochemical Co. Ltd.) was taken by microbalance in the precision instrument room and dissolved in 5 ml PBS (Wuhan Boster Biological Co. Ltd.) to form a mixed solution. Two 20 mL medical syringes were selected, one of which extracted the above-mixed solution and the other extracted 5 ml complete Freund's adjuvant (SIMGA), respectively, with medical tee connection on both ends of the syringe; the medical tee and syringe were buried in the ice basin, and the bolus injection was repeated for about 30–50 minutes, and finally an emulsion in oil was formed, and it was ensured that the emulsion in oil dripped into the water to gather and not disperse, which indicated the preparation of synthetic immunogen success. Then the successfully prepared synthetic immunogen was stored in a refrigerator at −4°C; within 12 hours of effective utilization time, it was applied, and repeated freezing and thawing was avoided.

#### 2.3.3. EAMG Model Establishment [15]

The anaesthetized mice were immunized 3 minutes later. In the model group, each mouse was given 50 *µ*L synthetic immunogen (including 50 *µ*g mouse peptide) in total 200 *µ*L at the bottom four parts of shoulders and hind feet, respectively. On day 1, mice were immunized with a synthetic immunogen containing complete Freund's adjuvant, and on days 30 and 50, mice were immunized with a synthetic immunogen containing incomplete Freund's adjuvant (SIMGA). Mice in the blank control group were injected with the same dose of normal saline at the same time and location. Model identification was performed on day 70 after the initial immunization.

#### 2.3.4. Model Identification

During the modeling process, the breathing, eating, exercise, posture, hair brightness, and other conditions of the mice were observed every other day, and the body weight was measured to make a body weight curve to compare the difference in weight change between the normal group and the model group. Muscle strength was measured, referring to the grading method of Lennon et al. [16]; the muscle strength of mice was divided into 4 levels: level 0, normal muscle strength, and no weakness, recorded as 0; level 1, limb muscle strength decline, movement reduction, and bite weakness, score 1; level 2, obvious weakness, tetraplegia, weakness, poor coordination of movement, and drooping head and tail, score 2; and grade 3, outstanding symptoms of muscle weakness, even worse difficulty breathing, and dying or death, score 3. The level of serum AChR-Ab was detected; blood was collected by the capillary method of the orbital venous plexus of mice, left standing at room temperature for 1 h, and then placed in a centrifuge for centrifugation, speed: 3,000 rpm, time limit: 10 min; and the serum was stored at 20°C for determination. Enzyme-linked immunosorbent assay (ELISA) was used to detect antibodies, and the operation was carried out in accordance with the requirements of the kit. *P/N* = OD(*λ*)450 nm serum to be tested/OD(*λ*)450 nm normal control serum. When P/N ≥ 2.1, AChR-Ab is positive.

#### 2.3.5. Treatment of EAMG Mice

After the model was successfully established, the mice were divided into five treatment groups: model group, mimic-NC group, miR-181a-mimic group, si-NC group, and si-TRIM9 group, each with 8 mice. Mice were injected with miR-181a-mimic, si-TRIM9 or miR-NC, and si-NC via intravenous (i.v.) tail vein. miR-181a-mimic and si-TRIM9 were synthesized through special chemical modification to increase their absorption into cells in the body and enhance or weaken their ability to resist RNase degradation. The dose was calculated as 80 mg/kg per mouse with three different injections. The clinical EAMG scores of each treatment group were measured every day after the first injection; mouse serum was collected; and the mice were sacrificed 21 days after treatment for further experiments.

### 2.4. Experimental Observation Indicators

#### 2.4.1. General Observation

After modeling group treatment, the weight change was also observed and recorded. The hair posture, gloss, appetite, activity, gait, breathing, and so on of each group of mice were observed. The clinical observations were scored according to the above-mentioned grading method of Lennon et al. [16].

#### 2.4.2. Real-Time Quantitative PCR

The TRizol method was used to extract total RNA from PBMCs and mouse serum and reverse transcription into cDNA using a reverse transcription kit (Japan TAKARA Company), conditions: 16°C for 30 minutes, 42°C for 30 minutes, and finally 80°C for 5 minutes. Real-time quantitative PCR was used for predenaturation at 95°C for 5 minutes, followed by 90°C for 15 s, 60°C for 15 s, and 72°C for 1 minute, for a total of 40 cycles. The experimental operation was carried out in strict accordance with the instructions of the corresponding kit, and the results were analyzed using the 2^−△△Ct^ method, where △Ct = Ct_target gene_ − Ct_control gene_. The serum miR-181a, TRIM9, U6, and GAPDH amplification primers were synthesized by Shanghai Shenggong Biological Engineering Co. Ltd. The primer sequences are shown in Table 1.

#### 2.4.3. Dual-Luciferase Report

The binding sites of miR-181a and TRIM9 were predicted and analyzed through the bioinformatics website (NECORI). The luciferase reporter method was used to verify the binding relationship between miR-181a and TRIM9. WT-TRIM9 plasmid and MUT-TRIM9 plasmid were constructed; Lipofectamine 2000 was used to transfect mimic-NC, miR-181a-mimic, WT-TRIM9, and MUT-TRIM9 into cells, 48h after transfection, The dual-luciferase report analysis kit was used to analyze the luciferase activity.

#### 2.4.4. Enzyme-Linked Immunosorbent Assay (ELISA)

The levels of IL-4, IL-6, and TNF-*α* in mouse serum were determined by enzyme ELISA. The standard wells and sample wells to be tested were marked on the microtiter plate, and 50 *μ*L of standards of different concentrations were added to the standard wells according to the sequence. The samples to be tested were numbered and labeled in order, and 10 *μ*L of the sample to be tested was added to the sample wells of the microtiter plate, and then 40 *μ*L of sample diluent was added, while the blank wells were not added. 100 *μ*L of HRP-labeled detection antigen was added to the standard and sample wells. Each well was fixed with a sealing film and incubated in a 37°C water bath for 60 minutes in a constant temperature box. Tear off the sealing film, pour out the liquid and spin dry, add washing liquid to each hole, let it stand for 30 seconds, and then pat dry. The whole process is repeated 5 times. 50 *μ*L of substrates A and B were added to each well and incubated at 37°C for 15 minutes in the dark. 50 *μ*L stop solution was added to each well to stop the reaction. Within 15 minutes, measure the OD value of each well on a 450 nm microplate reader and draw a standard curve.

### 2.5. Statistical Methods

SPSS21.0 software was used for analysis. The normality of measurement data was first tested. All indicators were expressed as mean ± standard deviation. When the mean comparison between two independent samples conformed to the normal distribution, t-test (homogeneity of variance) or approximate t-test (variance uneven) was used. The rank-sum test was used when the normal distribution was not met; single-factor analysis of variance was used for the comparison of sample means between multiple groups, and the LSD method was used for comparison between groups. Multiple groups of models were analyzed continuously at different time points, using variance analysis of repeated measurement data. *P* < 0.05 is considered statistically significant.

## 3. Results

### 3.1. Expression of miR-181a and TRIM9 in MG Patients

Detecting the expression of miR-181a and TRIM9 in MG patients, it was found that miR-181a was low in MG and TRIM9 was high in MG, both of which were statistically significant (*P* < 0.05; Figures 1(a) and 1(b)).

### 3.2. Establishment of the EAMG Model

There were a total of 45 mice in the model group who have the disease, and the success rate of modeling was about 72.58%. During the modeling period, 4 mice died successively, which may be caused by severe lung infection, death due to overanaesthesia, or operational errors. No mice died in the normal group. Before immunization, the body weight of C57BL/6 mice in the normal group and the model group was not statistically different. After immunization, the body weight of the C57BL/6 mice in the normal group and the model group increased. However, mice in the model group showed weakness, decreased dietary intake, and began to show a downward trend in body weight. Compared with the normal group, there was a significant statistical difference (*P* < 0.05; Figure 2(a)).

Observing the clinical symptoms of the mice, it was found that the mice in the normal group had a normal diet, were flexible in movement, and did not have a raised posture; the mice in the model group had a reduced diet, weak struggling strength, and slow movement. In terms of muscle weakness, the model group was significantly different from the normal group (*P* < 0.05). Serum AChR-Ab titer was detected. Compared with the normal group, the AChR-Ab titer level of mice in the model group was significantly increased, and there was a significant statistical difference (*P* < 0.05; Figures 2(b) and 2(c)).

### 3.3. Expression of miR-181a and TRIM9 and the Changes of Inflammatory Factors in the Serum of EAMG Model Mice

Analyzing the expression of miR-181a and TRIM9 and the changes of inflammatory factors in the serum of EAMG model mice, it was found that compared with the normal group, the expression of miR-181a in the serum of model group mice was reduced; the levels of TRIM9 and inflammatory factors IL-4, IL-6, and TNF-*α* increased, both of which were statistically significant (*P* < 0.05; Figures 3(a)–3(c)).

### 3.4. Effect of miR-181a on the Clinical Symptoms of EAMG Model Mice

To analyze the effect of miR-181a on the clinical symptoms of EAMG model mice, we upregulated the expression of miR-181a and found that compared with the model group, the changes of miR-181a in the mimic-NC group were not significant, while the expression of miR-181a in the mir-181a-mimic group was significantly increased (*P* < 0.05; Figure 4(a)). The observation of clinical symptoms showed that compared with the mimic-NC group, the clinical symptoms of the miR-181a-mimic group were improved, and the muscle weakness symptom score was decreased, with a significant statistical difference (*P* < 0.05; Figure 4(b)).

### 3.5. Effect of miR-181a on Inflammatory Factors in EAMG Model Mice

Analyzing the effects of miR-181a on inflammatory factors IL-4, IL-6, and TNF-*α* in EAMG model mice, it was found that the levels of IL-4, IL-6, and TNF-*α* in serum of miR-181a-mimic mice were significantly decreased, with statistical significance (*P* < 0.05; Figure 5).

### 3.6. miR-181a Can Target the Expression of TRIM9

To explore the relationship between miR-181a and TRIM9, we used the bioinformatics website (NECORI) to predict that the two have binding sites. The dual-luciferase report experiment showed that the luciferase activity of TRIM9-WT transfected with miR-181a-mimic decreased, while the luciferase activity of TRIM9-MUT transfected with miR-181a-mimic did not change significantly. It indicates that there is a targeting relationship between them (*P* < 0.05; Figure 6(a)). The serum TRIM9 of mice transfected with miR-181a-mimic was significantly decreased, and there was a statistical difference (*P* < 0.05; Figure 6(b)), These results suggest that miR-181a can target the expression of TRIM9.

### 3.7. Improvement Effect of TRIM9 on the Condition of EAMG Model Mice

To explore the effect of TRIM9 on the clinical symptoms of EAMG model mice, we interfered with the expression of TRIM9 and found that compared with the model group, TRIM9 in the si-NC group did not change significantly, and the expression of TRIM9 in the si-TRIM9 group was significantly decreased (*P* < 0.05; Figure 7(a)). Observing its clinical symptoms, it was found that compared with the si-NC group, the clinical symptoms of the si-TRIM9 group mice were improved, and the muscle weakness symptom score, and the levels of inflammatory factors IL-4, IL-6, and TNF-*α* were significantly reduced, with statistical significance (*P* < 0.05; Figures 7(b) and 7(c)).

## 4. Discussion

MG is a recognized autoimmune disease that affects signal transmission at the neuromuscular junction. In most patients with MG, the blockade of pathological antibodies blocks the nicotinic AChR at a part of the neuromuscular junction, resulting in that the neurotransmitter ACh cannot act on the corresponding receptor to perform physiological functions, thereby triggering the neuromuscular junction disorders of signal transmission function [17]. MG is currently the most recognized autoimmune disease of the nervous system, and it is also the most common type of neuromuscular junction disease. Although the pathophysiological mechanism of MG has been studied a lot, there are still many unknowns. Therefore, a better understanding of MG will bring great benefits to the research and treatment of this disease. Studies have detected changes in the spectrum of serum inflammatory factors and chemokines in MG patients, and it is speculated that these factors may be involved in the development of the disease [18]. Because the inflammatory environment plays a very important role in the development of this disease, appropriate interventions for inflammation are a very promising treatment strategy for future research.

Environmental factors have an important impact on the occurrence and development of diseases, which involve the process of the peripheral immune response. At present, multiple miRNAs have been confirmed to be involved in mediating the body's peripheral immune response, mainly through the toll-like receptor signaling pathway, involving mononuclear cells and macrophages [19]. In terms of treatment, the current research strategies for miRNAs focus on maintaining or inhibiting the function of a miRNA. A single miRNA can regulate its multiple targets to affect the entire conduction pathway, which provides the possibility for the treatment of diseases. It has been reported that miR-181a can regulate immune function and play a pivotal role in the innate and adaptive immune response [20]. miR-181a is also abnormally regulated in other autoimmune diseases, but its role in MG has not been studied in depth. The TRIM9 gene belongs to the three-domain protein family, which is found in all multicellular animals and currently contains more than 70 members. More and more evidence show that many TRIM family proteins are related to anti-infective immunity [21, 22]. Recently, it has been reported in the literature that TRIM9 is related to the regulation of the NF-KB signaling pathway [23]. We used the bioinformatics website to find that miR-181a has a binding site with TRIM9, so we discussed its related role in MG.

In our research, we found that in the PBMCs of MG patients and the serum of EAMG mice, the expression of miR-181a was downregulated, and the expression of TRIM9 was upregulated; the dual-luciferase report analyzed that miR-181a has a targeting relationship with TRIM9 and miR-181a can target the expression of TRIM9. It suggests that miR-181a and TRIM9 are related to the pathogenesis of MG. In order to explore the role of miR-181a and TRIM9 in MG, we established an EAMG mouse model. We observed that the mice in the model group lost weight, decreased diet, weak struggling strength, weak hissing, and slow movement. The score of myasthenia symptoms increased, and the serum AChR-Ab titer increased, confirming the successful establishment of model mice. We also observed that the serum levels of IL-4, IL-6, and TNF-*α* in EAMG mice were abnormally increased. It suggests that EAMG mice have a higher level of inflammation.

The cells are the main helper cells of the body, in which Th1 mainly secretes proinflammatory cells such as IL-2 interferon (IFN-*γ*) and tumor necrosis factor (TNF-*α β*) and activates cellular immunity by regulating hypersensitivity response and inflammation. Th2 cells secrete IL-4, IL-6, and other cytokines, regulate the growth and differentiation of B cells, counteract by inhibiting macrophages, play a synergistic effect with IFN-*γ*, assist AChR-specific B lymphocytes to proliferate and produce AchR-Ab, and initiate humoral immunity. The balance of the body's immune function is maintained by the regulation of cytokines secreted by Th1 and Th2 [24–26]. In this experiment, after upregulating miR-181a or interfering with TRIM9, serum miR-181a in EAMG mice was significantly upregulated; TRIM9 was significantly downregulated; its clinical symptoms were alleviated; and serum inflammatory factors IL-4, IL-6, and TNF-*α* levels were reduced. It is suggested that the regulation of miR-181a and TRIM9 can reduce the level of MG inflammatory factors and improve the symptoms of MG muscle weakness.

To sum up, in MG, miR-181a is lowly expressed, and TRIM9 is highly expressed; miR-181a can reduce the level of MG inflammatory factors through targeted regulation of TRIM9 expression and has the effect of improving the symptoms of MG. However, due to time and sample size, the relationship between miR-181a, TRIM9, and the clinical characteristics and prognosis of MG patients could not be discussed. Therefore, in follow-up studies, miR-181a, TRIM9, and different MGs can be discussed. The relationship between typed patients and prognosis provides epigenetic evidence and new development directions for the clinical treatment and pathogenesis of MG.

## Figures and Tables

**Figure 1:** Expression of miR-181a and TRIM9 in MG patients. Note: compared with healthy controls, ^*∗∗*^*P* < 0.01.

**Figure 2:** Identification of the EAMG model. Note: compared with the normal group, ^*∗*^*P* < 0.05.

**Figure 3:** Expression of miR-181a and TRIM9 and the changes of inflammatory factors in the serum of EAMG model mice. Note: compared with the normal group, ^*∗*^*P* < 0.05.

**Figure 4:** Effect of miR-181a on the clinical symptoms of EAMG model mice. Note: compared with mimic-NC group, ^*∗*^*P* < 0.05.

**Figure 5:** Effect of miR-181a on inflammatory factors in EAMG model mice. Note: compared with mimic-NC group, ^*∗*^*P* < 0.05.

**Figure 6:** miR-181a can target the expression of TRIM9. Note: compared with mimic-NC and mimic-NC groups, ^*∗*^*P* < 0.05.

**Figure 7:** Improvement effect of TRIM9 on the condition of EAMG model mice. Note: Compared with mimic-NC group, ^*∗*^*P* < 0.05.

**Table 1:** PCR primer sequence.

Name	Primer sequence
miR-181a	Forward (5'-3'): CTCAACTGGTGTCGTGGAGTCGGCAATTCAGTTGAGACTCAC
	Reverse (5'-3'): ACACTCCAGCTGGGAACA TTCAACGCTGTCG

U6	Forward (5'-3'): CTCGCTTCGGCAGCACA
	Reverse (5'-3'): AACGCTTCACGAATTTGCGT

TRIM9	Forward (5'-3'): CCCATGGAAGAGATGGAAGAAGAG
	Reverse (5'-3'): CTCACGGAGCTGGGGCTTGGGG

GAPDH	Forward (5'-3'): AGTATGACTCCACTCACG
	Reverse (5'-3'): GGTAGAAGGTCCTCGCTC

## Data Availability

The data used and analyzed during the current study are available from the first author and corresponding author on reasonable request.
